The article "A Multiagent Memetic Optimization Algorithm Based on Temporal Asymptotic Surprise in Complex Networks to Reveal the Structure of the Dynamic Community" was published in 2022. Journal: Comput Intell Neurosci.

# A Multiagent Memetic Optimization Algorithm Based on Temporal Asymptotic Surprise in Complex Networks to Reveal the Structure of the Dynamic Community

**DOI:** 10.1155/2022/6976875

**Published:** 2022-06-30

**Authors:** Somayeh Ranjkesh, Behrooz Masoumi, Seyyed Mohsen Hashemi

**Affiliations:** ^1^Department of Computer Engineering, Science and Research Branch, Islamic Azad University, Tehran, Iran; ^2^Faculty of Computer and Information Technology Engineering, Qazvin Branch, Islamic Azad University, Qazvin, Iran

## Abstract

Complex networks are used in a variety of applications. Revealing the structure of a community is one of the essential features of a network, during which remote communities are discovered in a complex network. In the real world, dynamic networks are evolving, and the problem of tracking and detecting communities at different time intervals is raised. We can use dynamic graphs to model these types of networks. This paper proposes a multiagent optimization memetic algorithm in complex networks to detect dynamic communities and calls it DYNMAMA (dynamic multiagent memetic algorithm). The temporal asymptotic surprise is used as an evaluation function of the algorithm. In the proposed algorithm, work is done on dynamic data. This algorithm does not need to specify the number of communities in advance and meets the time smoothing limit, and this applies to dynamic real-world and synthetic networks. The results of the performance of the evaluation function show that this proposed algorithm can find an optimal and more convergent solution compared to modern approaches.

## 1. Introduction

Dynamic networks change over time and are used in various fields. Identifying dynamic communities in complex networks is of great importance. A community in a complex network is a collection of close operations with other community entities. The existence of direct communication is a unique and essential action. Most of the new, improved tools and algorithms have been used for static networks, where the input graph cannot be changed, while most real networks have a dynamic nature [1]. Because real-world networks constantly change dynamically, community detection in static networks cannot capture natural phenomena and essential dynamics. Discovering communities in dynamic networks helps to find the laws of network evolution processes, which have been necessary for obtaining basic structural information in social [2–4] and biological systems [5, 6]. Evolution-based methods integrate communities and their evolution by simultaneously considering current and historical community structures in dynamic networks [7]. With increasing access to dynamic networks, the issue of detecting dynamic communities has become a new and vital topic in research, and various methods have been proposed for it [8, 9]. If static network-based methods identify real-world network communities, critical changing situations are easily lost [10]. Optimization has been considered the most critical issue in evolutionary sciences and methods. Evolutionary methods provide computational methods in which an iterative process is used to improve the resulting solutions until the termination condition is met.

The article "A Multiagent Memetic Optimization Algorithm Based on Temporal Asymptotic Surprise in Complex Networks to Reveal the Structure of the Dynamic Community" was published in 2022. Journal: Comput Intell Neurosci.

One of the optimization algorithms is an advanced discrete version of the Water Cycle Algorithm (WCA) to solve the Traveling Salesman Problem (TSP) [11]. A PSO-based optimization method is proposed for fuzzy navigation cognitive maps [12]. In this method, the complexity of the optimization problem requires the automatic adaptation of fuzzy cognitive map parameters, which evolutionary algorithms have proven to be effective in this field. Other optimization algorithms include a reinforcement learning-based control method that uses a Q-learning algorithm and meta-heuristic gravity search algorithm and has good performance to solve optimization problems [13]. An optimization method based on the heuristic algorithm is proposed in [14], which uses effective rule classification for string adaptation architectures with heterogeneous bit divisions. This method uses the uniqueness of the target pattern to classify all the characters in the target law and estimate the distance between strings to reduce memory demand. The optimization of fuzzy controllers for nonlinear processes is described in [15], which uses a meta-heuristic algorithm whose evaluation results indicate the high efficiency of this method.

The problem space on static problems remains unchanged during the optimization process. At the same time, most optimization problems are dynamic in the real world; the problem search space changes during the optimization process. In static optimization problems, finding the global optimal point is the primary goal, while finding the optimal global effectiveness is not the only goal of dynamic optimization. Tracking the optimal point in the problem space is very important. It is noteworthy that in many evolutionary optimization findings in dynamic environments, the concept of dynamic problems or time-dependent problems is not discernible. In these findings, dynamic optimization problems are defined sequentially as static problems. We have a dynamic problem using the time function in optimization; otherwise, we have a static problem [16]. In real-world network analysis, when data become temporal, the issue of modeling structural changes in networks becomes critical, and these types of networks become evolutionary. The activity of user groups over time can predict future behaviors on the network, such as clusters of famous writers in the Blogosphere [2], online networks such as Facebook and Twitter, and mobile networks. Dynamic networks have become widely popular in many fields and provide dynamic tracking of network structure [17]. In dynamic networks, two conflicting criteria are often considered for the problem of community recognition. First, they need to maximize the quality of the snapshot and measure the clustering performance of the photo at this time. Then, minimize time costs. In this way, in dynamic networks, the problem of community structure recognition can be considered a multiobjective optimization problem [18].

The article "A Multiagent Memetic Optimization Algorithm Based on Temporal Asymptotic Surprise in Complex Networks to Reveal the Structure of the Dynamic Community" was published in 2022. Journal: Comput Intell Neurosci.

In this paper, a new algorithm is introduced called a dynamic multiagent memetic algorithm in unweighted and undirected complex networks. In this algorithm, the agents are placed in a network-like structure. This algorithm is then used in complex networks for dynamic community detection and is named DYNMAMA (dynamic multiagent memetic algorithm). The evaluation function used in this algorithm for the dynamic environment is based on an example of an improved surprise function called temporal asymptotical surprise (TAS). The most popular criterion for the quality of a partition in a static network is modularity. However, this criterion is not a good choice in dynamic networks because the measurement has an inherent resolution limit. Surprise can overcome the resolution limit, and we can use it to reveal the exact community structure of complex networks. But surprise optimization has high computational complexity. We use the TAS formula in the structure of multiagent memetic algorithms in dynamic networks and conclude that it can achieve better results in detecting communities. We show that with this function, we can obtain better results in the problem of dynamic community detection, and we can apply it to other problems of the dynamic environment. DYNMAMA is suitable for handling large-scale complex problems.

In the following, the structure of the paper is as follows: in the second part, some related works are briefly reviewed. In the third part, dynamic community detection is explained. In the fourth section, optimization and multiagent systems are described. In the fifth part, a multiagent memetic optimization algorithm in complex networks for dynamic community detection is introduced. In the sixth part are the results of tests and evaluations. The seventh part includes discussion and future work, and the last part is the conclusion.

## 2. Related Works

The benefits of detecting communities in dynamic networks have led to much research in this area, such as methods based on two-step strategy [19], incremental clustering, evolutionary clustering [20], and multiagent algorithms [21]. We analyzed the structure of the distributed community through a tracking method. Another method is to use a few snapshots of the fixed network to evolve communities over time. It introduces a clustering method that tracks and evaluates the evolution of clusters, which are the same communities, over time.

The article "A Multiagent Memetic Optimization Algorithm Based on Temporal Asymptotic Surprise in Complex Networks to Reveal the Structure of the Dynamic Community" was published in 2022. Journal: Comput Intell Neurosci.

FacetNet, presented in [2], is a structure for community analysis in dynamic networks which operates based on instant photo cost optimization and ensures that it converges to an optimal local solution. Its convergence is slow, and communities must first be identified for each time slot and then compared to determine correspondence. The idea provides a framework for discovering communities that maximize temporal evolution. The concept of game theory has been used to identify static communities [20, 21]. This approach has also been proposed by Alvari et al. To identify communities in dynamic networks, the game theory method provides for dynamic community detection in which each node behaves as a logical representative [22]. Structures for evolutionary spectrum clustering are provided that include cluster quality maintenance parameters and cluster membership maintenance. In evolutionary clustering, we must take two goals into account: that the result of good clustering should be well-proportioned with current data and also not be significantly different from recent history at the same time. In this idea, smoothness measurement is integrated into the overall measure of clustering quality using the well-known k-means clustering. In [18], a multiobjective safety algorithm is presented. This algorithm can optimize both modularity criteria and normalized mutual information criteria simultaneously. A multiobjective method is proposed that identifies communities with temporal softness as a multiobjective problem and is based on genetic algorithms. The main advantage of this algorithm is that it automatically offers a solution that shows the best exchange between the obtained clustering accuracy and the deviation from one step to another [4]. A genetic algorithm with merging and splitting operators called MSGA [23] has been proposed to identify a dynamic community based on asymptotic surprise [24] and the maximum temporal asymptotic surprise to measure and calculate the quality of partitions in a dynamic network. Wang et al. [25] have proposed a new method of targeted optimization for community-based immunization to select immunization nodes. In this method, the structures of society are first discovered. Then, according to the characteristics that exist in the structure of society, potential candidates are limited. Finally, a new memetic algorithm selects safe nodes from the node set. Targeted immunization is formulated as an optimization problem. As mentioned earlier, dynamic communities change at different intervals and thus evolve with other developments. We can offer various approaches to achieve these communities [26]. One of these methods is the instant optimization that the currently identified associations should be the most relevant associations that only consider the current state of the network [27–29]. In the temporal trade-off method, the communities identified presently correspond to the balance between the best relatively stable communities to the network and the history of the communities built. This method consists of three steps. First, identify fixed communities at present. Second, identify existing communities later, using communities acquired earlier, and in the third step, it returns to the second step to complete all the processes. In the cross-time community detection method, all stages of evolution are studied simultaneously. By considering in a single transition all network cycles and creating a single decomposition, single community detection is performed, i.e., instant detection on all snapshots [30–34].  Figure 1 shows some of the most prominent algorithms that have been proposed so far for these approaches. Various ideas of the memetic algorithm have been proposed for community detection in a static environment.

The article "A Multiagent Memetic Optimization Algorithm Based on Temporal Asymptotic Surprise in Complex Networks to Reveal the Structure of the Dynamic Community" was published in 2022. Journal: Comput Intell Neurosci.

The memetic algorithms have been able to attract the interest of many researchers and are one of the most desirable methods of evolutionary optimization.  Table 1 shows examples of the application of memetic algorithms in community detection in networks, which shows the type of crossover operators and mutations used in them. Several studies focused on the neighbor mutation that guarantees that each mutated gene is linked only with one of its neighbors. This method can cause one of two effects that relate to a community's state by either splitting a single community or combining two communities and ultimately modifying the community structure.

In adaptive mutation, the mutation rate varies according to the fitness value, previous mutation rate, or the number of generations (assuming that the mutation points are determined randomly). Other new methods have been proposed in dynamic networks to solve and optimize the problem of community detection.

Mishra et al. [45] proposed a tree-based structure in dynamic networks that uses connection and penetration methods to maintain and record information about the discovery and change of communities at different time intervals. The spiderweb method is suggested in [46], which uses the idea of a spider web by forming subgraphs of nodes to identify a community. In [47], a new method for identifying dynamic communities is introduced, which works based on the distance between the resistance, identifying the core node, and using a noise community. Also, a method based on classification approaches, including top-up, top-down, and based on the data structure to identify the community in dynamic networks, is proposed [48]. Other new algorithms based on ant colony and network node attributes have been proposed in [49, 50] for community detection.

The article "A Multiagent Memetic Optimization Algorithm Based on Temporal Asymptotic Surprise in Complex Networks to Reveal the Structure of the Dynamic Community" was published in 2022. Journal: Comput Intell Neurosci.

The chaotic memetic algorithm is a new method for detecting the structure of the community in complex networks that use a modularity function [51]. In this method, a chaotic memetic algorithm is proposed that uses both chaotic numbers instead of random numbers in global and local search processes, preserving population diversity and preventing local optimization from falling.

## 3. Dynamic Community Detection

Community detection, one of the problems of social network analysis, is the detection of hidden structures in the network and the division of the network into partitions where the communication between network members is dense in each section. Network partitioning is modeled in the form of the objective function optimization problem. Detecting communities fall into the category of NP-Hard issues.  Figure 2 shows the relationship of members of a community.

Community detection is often used in complex networks. These networks represent systems or data that are not random and can originate from nature, community, or anything else. A group of nodes can be defined as an association in a network whose dense internal connections rarely have external links. We can obtain commonalities or relationships from community detection [52]. Today, networks are extensive in scales that are constantly changing their structure. A dynamic network can be considered a collection that includes snapshots at different time intervals. The first feature of dynamic community detection is used in dynamic networks. Networks evolve and can originate from a variety of contexts. Gathering information in real time as soon as they appear is another way to get a changing network.

We can obtain the community model by combining a previous timestamp or a network snapshot. According to a dynamic *G* network, periods can be discrete or continuous in a dynamic community without changing the nature of dynamic communities. We can use operations in dynamic communities that include six different operations on communities. Cazabet et al. [53] added a seventh operation, which provides for growth, contraction, merging, splitting, birth, death, and resurgence as shown in Figure 3. Figure 3 shows that the growth operation can enlarge a community by merging new nodes. The contraction operator in a community means removing some nodes and making that community smaller. The merging operator involves combining two or more communities into one community. The splitting operator implies that a community can be divided into two or more other communities. In birth operations, we can create a new community over some time. The death operator means that a community can be destroyed or disappear at any time. In resurgence operations, a community that has vanished in a limited time can reappear at another time.

The article "A Multiagent Memetic Optimization Algorithm Based on Temporal Asymptotic Surprise in Complex Networks to Reveal the Structure of the Dynamic Community" was published in 2022. Journal: Comput Intell Neurosci.

Most optimization problems are dynamic in the real world, and the problem search space changes during the optimization process. Finding the global optimal point is not the only goal of dynamic optimization, and tracking the optimal point in the problem space is very important. If the cost function of the optimization problem is not a function of time, we are dealing with a static optimization problem. Still, if time also enters the cost function, the problem of optimization becomes dynamic. Effective optimization over time depends on the increasing effect of instabilities caused by the parameter space on the time vector. Complex time-dependent systems can have dense components in cohesive groups of nodes known as “communities.” In the real world, network topologies change over time. Figures 4 and 5 show the structure of a variable community with time, and the following figures show the evolution of the community in a dynamic network [54]. An evolutionary algorithm based on clustering in dynamic networks has been proposed by Chen et al. [55]. Other algorithms for detecting dynamic communities have also been proposed in [56–59].

## 4. Optimization and Multiagent Systems

The goal of optimization is to find the best acceptable answer, given the limitations and needs of the problem. There may be different answers to a problem, and the objective function is defined to select the optimal solution. Multiagent systems provide the opportunity to calculate and optimize many complex problems. There are two critical issues involved in designing multiagent systems: the first is the design of the agent, and the second is the creation of the environment for the performance and relationship between the agents, in agent design, how to build an agent capable of performing independent tasks and autonomous actions. In designing a community or operating environment, the key is how to create agents that can interact with one another. This relationship implies cooperation, coordination, and negotiation between agents. It is indispensable for accomplishing the tasks we have been given because not all agents have common goals or create the same interests. In Figure 6, you can see the structure of an environment with two agents and what parts each agent contains, and what kind of relationship it has with the other agent. Their neighborhood knowledge determines the relationship between the two agents. They were deciding whether two agents were adjacent to each other.

The article "A Multiagent Memetic Optimization Algorithm Based on Temporal Asymptotic Surprise in Complex Networks to Reveal the Structure of the Dynamic Community" was published in 2022. Journal: Comput Intell Neurosci.

We can combine multiagent systems and evolutionary algorithms to form new algorithms to solve optimization problems. The optimization algorithm is introduced that uses the structure of a multiagent system to optimize the extractive text summarization problem [60]. This method combines the optimization algorithm based on biogeography (BBO) and the concepts of multiagent systems to create an optimal summary, the results of which show the efficiency of this method. Agents live in a network, and each agent is fixed at a network point. All agents can increase their energy in competition with their neighbors and use domain knowledge. Combining evolutionary algorithms and multiagent systems leads to convergence to optimal global solutions, which occurs at high speed. They are also used to solve large-scale problems with thousands of dimensions, and this hybrid structure has been able to achieve good performance and reduce computational costs. Also, a method based on the multiagent particle swarm optimization approach has been proposed to improve the text summarization. In this method, each particle is upgraded with the status of multiagent systems [61]. The environment, as an agent, provides environmental information to other agents. When the search is limited to points that have not yet been met, the search speed increases.

In the community detection problem, the agent is defined as dividing a network, a candidate solution to solve the problem. Because the agents live in a network-like environment, they are called network agents who can exchange information with their neighbors. Multiagent systems have been integrated with evolutionary algorithms to solve constraint satisfaction problems and combinatorial optimization problems with satisfactory results.

## 5. Multiagent Memetic Optimization Algorithm to Dynamic Community Detection (DYNMAMA)

The memetic algorithm is one of the evolutionary algorithms, and it is a hybrid optimization method that adds local search to the evolutionary optimization process, increases convergence speed, and can successfully solve complex optimization problems. In this algorithm, each member of the population can grow its fitness as its neighbors. The utility of each of the answers in this algorithm is calculated based on the fitness function, and it generates new responses using the intersection and mutation operators. A local search is done on each generation at the end of this algorithm. A set of solutions of that generation and a subset of the current generation are transferred for the next generation's survival. Generating new generations continues until fulfilling the stop condition. The local search strategy is the most critical key to the effectiveness of memetic algorithms.

The article "A Multiagent Memetic Optimization Algorithm Based on Temporal Asymptotic Surprise in Complex Networks to Reveal the Structure of the Dynamic Community" was published in 2022. Journal: Comput Intell Neurosci.

The proposed algorithm, the multiagent memetic algorithm in dynamic community detection, is called DYNMAMA. In this structure, agents live in a network-like environment. Agents can live in the environment and apply activities according to their understanding, and specific goals can guide them. Because each agent interacts with its environment and other agents, it can increase its energy, which allows the multiagent memetic algorithm to optimize the objective function value. We can base agents' decision-making on parameters defined as agents' input, and agents can use appropriate actions and activities to solve and optimize the problem. One of the most critical applications of multiagent systems is modeling complex systems, and the structure of networks can be considered a complex system. We can use graphs for modeling that graph nodes are agents, and having a link and edge between agents means having their relationship. Multiagent systems can be the optimal way to solve the problem of complexity in the structure of networks such as social networks. If we want to model complex dynamic networks, this is very costly and requires a lot of processing. We can model this complex dynamic network with less cost and processing because of agents' features in multiagent systems, such as scalability and flexibility. An agent can use local search to increase the value of its evaluation function based on the appropriateness of the importance of its neighbor's evaluation function. When the environment of multiagent systems is dynamic, then for learning operations, we must constantly update agents. Sharing knowledge between agents and their neighbors leads to joint learning, effectively removing and reducing obstacles. Each agent competes or cooperates with other neighboring agents to achieve its ultimate goal in optimization issues. Neighborhood competition, crossover, mutation, and self-learning operators are defined for these operating behaviors.  Figure 7 introduces the parameters that make up our proposed algorithm and explain how we can apply the parameters according to the application of the algorithm. In the proposed algorithm, we need to enter the data at each step for processing.

The article "A Multiagent Memetic Optimization Algorithm Based on Temporal Asymptotic Surprise in Complex Networks to Reveal the Structure of the Dynamic Community" was published in 2022. Journal: Comput Intell Neurosci.

Initialization should be done based on the data of that time and based on the number of nodes and connections between nodes, then partitioning should be done, and we should enter the next stage or time. We will enter new data into the program again and operate the data again. This method does not need to specify the number of communities in advance and, at the same time, satisfies the time smoothing limit. The initial values of the agents are random, and in the following steps, the populations are randomly assigned with the best sample of the community in the previous time step. The dynamic network *G* is represented by a set of instantaneous images of the network *G*={*G*_1_,  *G*_2_,…,  *G*_*T*_) at time intervals  *T*.

DYNMAMA uses a locus-based adjacency encoding schema. This schema brings to these approaches the advantage that the number of communities does not need to be specified in advance. In this graph-based structure, each *g* genotype contains *n* genes. Each *g*_*i*_ gene can take up any of the neighboring node nodes. Therefore, any value of *j* assigned to the gene *i* is interpreted as a link between *i* and  *j*. As a result, these nodes are in the same community. For example, suppose a network is assumed to be in Figure 8. This graph has 15 nodes and can be divided into three communities. An example of a possible chromosome is illustrated. Each community is a subset of network vertices. The complex multiagent memetic algorithm for community detection has the following basic steps: neighborhood-based integration operator, hybrid integration operator, adaptive mutation operator, self-learning operator, fitness function, and local search, which are detailed in each step. Each of these parameters is described below.

### 5.1. Division Operator and Neighborhood Competition Based Integration (Split and Merging)

We consider the agent in the  *a*, *b* coordinates of the grid to be *Z*_*a*,*b*_, and the agent with the highest energy among the neighbors to be Max_*a*,*b*_. If the amount of energy *Z*_*a*,*b*_ is greater than the amount of energy Max_*a*,*b*_, then *Z*_*a*,*b*_ will be the winner, and it is one of the best and can survive; otherwise, the agent *Z*_*a*,*b*_ is replaced by Max_*a*,*b*_.

For the loser and replacement mode, two strategies can be proposed that emphasize exploitation or exploration Max_*a*,*b*_ chooses one of these strategies considering the probability. An agent locates at (*a*,  *b*), *a*,  *b* = {1,  2 …  Size}, and an agent *Z*_*a*,*b*_ consists of *N* genes. If there is a connection between nodes *i* and  *k*, then the  *g*_*i*_ gene takes the value of *k*. In this display, *k*=(*g*_*i*_=*k*) and the indices of *i* and *k* are in a similar community. We define a genotype that explores the relationship between specific nodes and communities. In this method, we consider two approaches to detect the allele value of a random gene from each agent. The gene selected for each agent that is randomly determined is called the target gene. We choose an approach by choosing a random number. We compare the energy of the modified energy agent(*Z*_*a*,*b*_) with the point of the best agent in the energy neighborhood Max_*a*,*b*_, and if the energy improves, we save the new agent. The modified agent (*Z*_*a*,*b*_) is compared with the energy of the best agent in its neighborhood (max_*a*,*b*_). In the case of energy improvement, the new agent is saved; otherwise, we will replace it with the best neighbor. If *Z*_*a*,*b*_ satisfies equation (1), it is a winner; otherwise, it is a loser.

(1) $$\begin{array}{c} \text{Energy }\left(Z_{a,b}\right)>\text{Energy}\left({\text{Max}}_{\text{a,b}}\right). \end{array}$$

Max_*a*,*b*_ is first mapped on [0,  1] and generates a new agent, New_*a*,*b*_, and then, New_*a*,*b*_ is put on the lattice point. We used the division and integration operator to remove lower energy agents from the network.

The article "A Multiagent Memetic Optimization Algorithm Based on Temporal Asymptotic Surprise in Complex Networks to Reveal the Structure of the Dynamic Community" was published in 2022. Journal: Comput Intell Neurosci.

### 5.2. Hybrid Integration Operator (Crossover)

In the proposed method, a neighboring integration operator is defined that consists of combining two types of two-point and uniform integrations. In this function, using two integration action strategies, an agent *Z*_*a*,*b*_ is integrated with the best agent in its neighborhood max_*a*,*b*_. Each strategy is selected based on the *P*_*x*_ probability. If *u*(0,1) < *p*_*x*_, the first strategy is adopted; otherwise, we will use the second strategy. The first strategy begins with the two-point integration and the random selection of points *k*_1_ and *k*_2_. If *u*(0,1) < 0.5, the genes between the two selected points of max_*a*,*b*_ are replaced with *Z*_*a*,*b*_; otherwise, we will replace the genes outside these selectable points with each other. In fact, in the first strategy, we map the genes between positions *k*_1_ and *k*_2_ of max_*a*,*b*_ to  *Z*_*a*,*b*_. Otherwise, the rest of the genes are mapped to  *Z*_*a*,*b*_. In the second strategy, a uniform integration operator is used in which max_*a*,*b*_ and  *Z*_*a*,*b*_ are integrated, and  *Z*_*a*,*b*_ is replaced with the new agent.

### 5.3. Mutation Operator

The mutation is performed based on the probability *p*_*b*_. If *u*(0,1) < *p*_*b*_, then the value of the gene is replaced by the neighbor allele's value in its neighborhood list. Also, the *p*_*b*_ changes to achieve better results in an adaptive mutation operator. Equation (2) shows the mutation.

(2) $$\begin{array}{c} P_{b^{\prime }}=\left(\frac{t}{N_{x}}+1\right)P_{b}, \end{array}$$

where *N*_*x*_ is the end criterion and  *P*_*b*_ is the probability of mutation.

The article "A Multiagent Memetic Optimization Algorithm Based on Temporal Asymptotic Surprise in Complex Networks to Reveal the Structure of the Dynamic Community" was published in 2022. Journal: Comput Intell Neurosci.

### 5.4. Local Search

The local search is applied to agents after generating a new generation and replacing it with previous generations in the proposed algorithm. Accordingly, for each agent, a neighborhood radius is considered that the neighbors of each agent *Z*_*a*,*b*_ in the proposed method are determined based on equation (3). Each agent is compared with the neighboring agents in terms of energy. In equation (3), *Z*_size_ is the size of the population. Agents are used to detect communities within graphs. We show the neighborhood structure we used in Figure 9.

(3) $$\begin{array}{c} {\text{neighbors}}_{a,b}=\left\{Z_{a^{\prime },b}\;,\;Z_{a,b^{\prime }},Z_{a,b^{\prime \prime }},Z_{a^{\prime \prime },b}\right\},\\ a^{\prime }=\left\{\begin{array}{cc} a-1, & a\neq 1,\\ Z_{\text{size}}, & a=1, \end{array}\right.\;a^{\prime \prime }=\left\{\begin{array}{cc} a+1, & \;a\neq Z_{\text{size}},\\ 1, & \;a=Z_{\text{size}}, \end{array}\right.\;\\ b^{\prime }=\left\{\begin{array}{cc} b-1, & \;b\neq 1,\\ Z_{\text{size}}, & b=1, \end{array}\right.\;b^{\prime \prime }=\left\{\begin{array}{cc} b+1, & b\neq Z_{\text{size}},\\ 1, & b=Z_{\text{size}}. \end{array}\right. \end{array}$$

### 5.5. Self-Learning Operator

In the proposed method, a network of small-scale *s* *Z* agents with the size *s* *Z*_size_ × *s* *Z*_size_ is created based on equation (4). In the following equation, *Z*_size_ is the size of the population.

(4) $$\begin{array}{c} sZ=\left\{\begin{array}{cc} Z_{a,b}, & a^{\prime }=1\;,\;b^{\prime }=1,\\ sZ_{a^{\prime },b^{\prime }}, & \text{otherwise}. \end{array}\right. \end{array}$$

*sZ*_*a*′,*b*′_ is created based on the neighborhood-based mutation operator on *Z*_*a*,*b*_ The split and merge operation improves agent energy until no improvement is achieved. The self-learning operator is essential in improving the performance of our proposed algorithm.

### 5.6. Fitness Function

A statistical measure of the community is called a surprise. The formula of this criterion is shown in the following equation:

(5) $$\begin{array}{c} S=-\text{ln}\overset{\text{min}\left(m,\;M_{\text{int}}\right)}{\underset{j=m_{\text{int}}}{\sum }}\frac{\left(\begin{array}{c} M_{\text{int}}\\ j \end{array}\right)\left(\begin{array}{c} M-M_{\text{int}}\\ m-j \end{array}\right)}{\left(\begin{array}{c} M\\ m \end{array}\right)}, \end{array}$$

where

- *M* = the maximal number of links
- *M*_int_ = the maximal number of intracommunity links
- *m* = the number of existing links
- *m*_int_  = the number of existing intracommunity links

Surprise can eliminate the degree of resolution and, by maximizing it, can accurately reveal the community structure of networks, but optimization with this method has high computational complexity. Trag et al. presented an exact asymptotic approximation of surprise or asymptotic surprise called asymmetric surprise or AS. Asymmetric surprise can accurately measure and quickly calculate the quality of partitions in a dynamic network. Detecting a dynamic community is a matter of maximizing this function. This method lacks a resolution that makes the structure of the community more accurate. Its formula is shown in the following equation:

(6) $$\begin{array}{c} S\approx m\left(q\;\log\frac{q}{q}+\left(1-q\right)\log\frac{1-q}{1-q}\right)=m\;D\left(q\mathrm{||}\left.\bar{q}\right.\right), \end{array}$$

where

- *q* = *m*_int_*/m*
- $\bar{q}$ = Mint/*M*
- *D*(*x*||*y*) is the KL divergence

Asymmetric surprise has been developed for the temporal asymptotical surprise (TAS) for dynamic community detection. We used TAS as the fitness function to optimize. For a given partition  *π*, the temporal asymptotical surprise at time *t*  is defined according to equation (7), which shows that the asymmetric temporal surprise at time *t* depends on AS at *t*,  *t* − 1,…,  *t* − *k*( 1 ≤ *k* ≤ *t* − 1). Given a partition *π*, we can obtain the total numbers of internal links *mint* and possible internal links *Mint*.

(7) $$\begin{array}{c} \text{TAS}\left(\pi ,G,t\right)=\left\{\begin{array}{cc} AS\left(\pi ,G_{1}\right), & t=1,\\ \beta .AS\left(\pi ,G_{t}\right)+\left(1-\beta \right).AS\left(\pi ,G_{t-1}\right), & t=2,3,\ldots ,T. \end{array}\right.. \end{array}$$

A chromosome is decoded into a partition, and the TAS associated with the partition and current time step is calculated using equation (7).

The article "A Multiagent Memetic Optimization Algorithm Based on Temporal Asymptotic Surprise in Complex Networks to Reveal the Structure of the Dynamic Community" was published in 2022. Journal: Comput Intell Neurosci.

A dynamic network  *G* is given by a series of network snapshots,  *G* = {*G*1,  *G*2,  . . . ,  *GT*}. Parameter *β* is an input parameter that measures the relative importance of the snapshot cost in the whole one. Therefore, to calculate the fitness of each population, first, the populations are converted to partition by decoding. Then, the fitness value for each population is calculated by the TAS function. If we consider TAS as a qualitative criterion for communities, the problem of detecting the structure of the community becomes the problem of finding the partition of the network with the optimal value of TAS. Algorithm 1 shows our proposed method, DYNMAMA, for dynamic community detection. We use TAS as an effective measure to evaluate the quality of a partition on the snapshot of the dynamic network. As an extension of asymptotic surprise, TAS is preferable for dynamic community detection because it can break resolution limits and supports temporal smoothness for adjacent snapshots.  Figure 10 shows the flowchart of the multiagent memetic algorithm in dynamic community detection, DYNMAMA. The value of parameters used in our proposed algorithm is according to Table 2.

## 6. Test Results and Analysis

In this section, we test the results of evaluating the effectiveness of using the multiagent memetic algorithm in complex networks for dynamic community detection (DYNMAMA). The results of the suitability value or the same TAS and NMI (normalized mutual information) [62] are calculated at each time step. As an evolutionary method, we have to set several parameters. Finally, we compare the proposed method with state-of-the-art approaches, such as MSGA [23], DYNMOGA [4], ESPRA [63], and FacetNet algorithms [2], which are well-known evolutionary approaches for the accurate detection of dynamic communities in networks. These methods are in dynamic networks and are based on evolution, which integrate the extraction and evolution of societies by simultaneously considering the structures of current and historical community. In MSGA, a genetic algorithm improved by the split and merge operator is used for dynamic community detection. First, the algorithm gets the dynamic network, the number of time steps, and the population size. Then, it generates the best partition for each time step. The initialization is divided into two parts. 90% of the initial populations are randomly selected, and the remaining 10% are quantified by the best samples of the previous population. The standard parameters are considered the same for better comparison in both methods.

In fact, by comparing this algorithm with our proposed method, we want to examine whether local search in a memetic algorithm can improve the results or not. In the DYNMOGA algorithm, which is based on a genetic algorithm, the discovery of communities in dynamic networks has been proposed as a multiobjective optimization problem to increase the quality of snapshots and reduce time costs. ESPRA is a clustering method for finding dynamic communities presented under temporal smoothness. FacetNet uses a random model to generate communities and a probabilistic model to capture community change and discovers communities that maximize time evolution. We run our algorithm in MATLAB 2016, and we select solutions with the maximum value of NMI at each run.

The article "A Multiagent Memetic Optimization Algorithm Based on Temporal Asymptotic Surprise in Complex Networks to Reveal the Structure of the Dynamic Community" was published in 2022. Journal: Comput Intell Neurosci.

### 6.1. Data Sets

We tested DYNMAMA performance on real-world dynamic networks and synthetic networks, which we describe below:

#### 6.1.1. Real-World Network: Enron Email

The data set used a collection of emails sent between employees of an organization collected between 1999 and 2002. The data set we reviewed is part of these emails sent to employees within the organization for 12 months. The smaller version of this data set contains the following: the number of employees is 151, and the number of emails sent is 50,572. Therefore, in the network structure, the number of 151 nodes and the number of directional links equal the number of emails sent. The Enron email data supporting this study's findings are available with the identifier “https://doi.org/10.1109/TKDE.2013.131” [4]. The number of different links without repetition is equal to 2235. Also, the number of time steps is 12.

#### 6.1.2. Synthetic Network: LFR Benchmark

This database is one of the standard graphs that achieve heterogeneity in the distribution of node degree and size of the community in the dynamic environment. The LFR data supporting this study's findings are available with the identifier [3]. That is, we can trace communities over time in unstable networks. This data set is a network generator that can generate dynamic network instances that include growth, contraction, merging, splitting, birth, death, and alternating communities. Each network consisted of 1000 nodes. Nodes have an average degree of 20, a maximum degree of 40, and a mixing parameter value of *μ* = 0.2 that controls the level of edges between communities. We set the power exponents for degree and community size to −1 and −2, respectively.

### 6.2. Evaluate the Quality of the Communities Detected

Communities detected by the proposed algorithms are analyzed using the NMI evaluation criterion. NMI determines the proximity of communities resulting from the proposed system to optimal communities. *A* and *B* are partitions of a network. If *A* and *B* are the same, *NMI*(*A*,  *B*)=1, and if *A* and *B* are entirely different, *NMI*(*A*,  *B*)=0. The definition of *NMI*(*A*,  *B*) is shown in the following equation:

(8) $$\begin{array}{c} \text{NMI}\left(A,B\right)=\frac{-2\sum_{i=1}^{k_{A}}\sum_{j=1}^{k_{B}}D_{ij\;}\log\left(D_{ij\;}N/D_{i.}D_{.j}\right)}{\sum_{i=1}^{k_{A}}D_{i.}\log\left(D_{i.}/N\right)+\sum_{j=1}^{k_{B}}D_{.j}\log\left(D_{.j}/N\right)}, \end{array}$$

where *k*_*A*_ is the number of communities in  *A*, *k*_*B*_ is the number of communities in *B*, *D* is the confusion matrix, and *N* is the number of elements.

In addition to NMI, the error rate [2] can also be used to evaluate the distance between a detected partition and the ground truth. At the error rate, the *Z* matrix is used to represent the partitions and the *G* matrix is used to represent the ground truth. If the number of nodes in the network is  *n*, the number of communities in a detected partition is  *k*, and the actual number of communities is  *m*,  *Z*=*n* × *k*, and  *G*=*n* × *m*. The error rate is then defined as the norm  *ZZ*^*T*^ − *GG*^*T*^, that is, nonzero inputs and the detected partition will be more accurate if the error rate is lower. The error rate measures the distance between the community structures represented by *Z* and *G*.

The article "A Multiagent Memetic Optimization Algorithm Based on Temporal Asymptotic Surprise in Complex Networks to Reveal the Structure of the Dynamic Community" was published in 2022. Journal: Comput Intell Neurosci.

### 6.3. Results of the DYNMAMA

First, the results based on the best NMI values in the Enron email network are presented for comparison and analysis. To calculate the NMI value, we need to know the initial communities in the Enron email network.  Figure 11 shows the NMI results for DYNMAMA, MSGA, DYNMOGA, and ESPRA. As you can see in Figure 11, our proposed method, DYNMAMA, has been more successful than other methods in obtaining values close to 1, which indicates the high accuracy of the proposed method and the high quality of the dynamic communities discovered. The MSGA algorithm has also obtained good values close to our proposed method. For example, in step 9, the NMI values obtained by DYNMAMA and MSGA are 0.8309 and 0.8024, respectively, which are close to each other. At this time, the NMI values obtained from the other two methods, DYNMOGA and ESPRA, are 0.6718 and 0.5491, respectively, which have weaker answers than our proposed method. Our proposed method maintains the NMI values obtained in these 12 time steps between 0.7625 and 0.8685. The highest value that the MSGA method has been able to get for NMI is 0.8081 in time step 3, for the DYNMOGA method, 0.7821 in time step 7, and for the ESPRA method 0.6527 in time step 10 in the Enron email network data set. In Figure 11, the lower error rate is related to our proposed algorithm in all time steps, which, for example, in step 6 was able to achieve the value of 508. The lowest error rates for other comparable algorithms are 610, 903, and 990 for MSGA, DYNMOGA, and ESPRA, respectively. We observe that in this network, the highest error rate in all time steps is related to the ESPRA algorithm.

In Table 3, the results of the TAS value in each time step are calculated for the best partitioning in each step in the proposed dynamic community detection algorithm, DYNMAMA, in the Enron email network. In other words, after determining the best solution or the best partition in each step, its TAS value is determined and shown in Table 3. Both DYNMAMA and MSGA methods use the TAS evaluation function, and the DYNMOGA method uses the *Q* modularity evaluation function. |*C*|_*D*1_ and |*C*|_*D*2_ are the number of dynamic communities detected in DYNMAMA and DYNMOGA methods, respectively, and |*C*|_*M*_ is the number of dynamic communities detected in MSGA. |*V*| and |*E*| are the number of nodes and edges, and |*E*^*∗*^| is the number of undirected edges.

The article "A Multiagent Memetic Optimization Algorithm Based on Temporal Asymptotic Surprise in Complex Networks to Reveal the Structure of the Dynamic Community" was published in 2022. Journal: Comput Intell Neurosci.

As shown in Table 3, the number of evaluation functions and the number of dynamic communities detected are variable at each time step for each method. For example, in time step 2, the numbers of dynamic communities obtained by the DYNMAMA method equal 12. For the two methods, MSGA and DYNMOGA are equal to 11 and 9, respectively. Also, at the same time step, the value of TAS in the DYNMAMA method is equal to 179.563, and in the MSGA method, it is equal to 178.376, and the value of modularity function in the DYNMOGA method is equal to 0.5348. In time step 12, the numbers of dynamic communities obtained by the DYNMAMA method are equal to 14, and for the two methods, MSGA and DYNMOGA are equal to 13 and 9, respectively. Also, at the same time step, the value of TAS in the DYNMAMA method is equal to 376.025, and in the MSGA method it, is equal to 329.668, and the value of modularity function in the DYNMOGA method is equal to 0.5175. In other words, the proposed method has been able to increase and improve the value of its evaluation function and detect more dynamic communities. Because both DYNMAMA and MSGA methods use the TAS function, their values at each time step for comparison are shown in Figure 12. As can be seen in the results, the proposed method (DYNMAMA) in the Enron email network has been able to achieve better results than the MSGA method and achieve better answers in each step. It allows for better partitioning, and the detected communities are more accurate. The structure of the communities detected by the proposed DYNMAMA method at time steps 3 and 4 for the email network can be seen in Table 4. If we want to compare operations in the third and fourth time steps according to Table 4, we see that, for example, in community number 1 of the third time step, nodes 1, 2, 6, 18, 22, 30, 31, 40, 49, and 75 have a membership in this community. We see that in the fourth stage, nodes 18, 30, 31, and 40 have lost their membership in community one and have joined community numbers 4, 10, 2, and 8, respectively. The number of detected communities has reached 16 in the third step and 13 in the fourth step.

The results of the LFR data set are shown below. We mentioned earlier that this benchmark is closer to real-world networks regarding node degrees and community size.  Figure 13 shows the performance of our proposed algorithm, DYNMAMA, and the other four algorithms, MSGA, DYNMOGA, ESPRA, and FacetNet, in the birth and death of the LFR network. In evaluating and comparing the results, we can see that the DYNMAMA method has obtained the NMI value always better than the other four methods and the value of 1 or relatively close to 1.

The article "A Multiagent Memetic Optimization Algorithm Based on Temporal Asymptotic Surprise in Complex Networks to Reveal the Structure of the Dynamic Community" was published in 2022. Journal: Comput Intell Neurosci.

The minimum NMI in the DYNMAMA method is 0.9967 in time interval 1. It means that our proposed method has always been able to obtain more accurate quality communities in periods of 1 to 10 than the other two methods.

The existence of local search in the structure of memetic algorithm and cooperation and evolution of factors in the network structure such as multiagents in the DYNMAMA method have improved the results continuously upward. DYMAMA and MSGA are relatively equal and close to each other in the birth and death part of the LFR data set at time intervals 2, 5, 7, and 8. DYNMOGA maintained the NMI values obtained, except for step one, between 0.9754 and 0.9936 in steps 2 to 10. ESPRA received the highest NMI value in time 5 with 0.9871. FacetNet also got the highest value in time 6 with 0.9878 and the lowest value in time 1 with 0.9714. In Figure 13, the lower error rate is related to our proposed algorithm in all time steps, which, for example, in step 6 was able to achieve the value of 69. The lowest error rates for other comparable algorithms are 84, 468, 2032, and 6543 for MSGA, DYNMOGA, ESPRA, and FacetNet, respectively. We observe that in this network, the highest error rate in all time steps is related to the FacetNet algorithm.

Figure 14 shows the performance of our proposed algorithm, DYNMAMA, and the four comparable algorithms in the expansion and contraction section of the LFR data set in 10 time steps. Both DYNMAMA and MSGA algorithms perform well. In each time step, DYNMAMA has higher accuracy in terms of NMI value in this part of the network than the LFR database, and except for time steps 2, 6, and 9, it has been able to obtain a value of 1 at other times. MSGA has also been able to get values close to 1, and the minimum NMI value for it in the time interval is four and equal to the value of 0.9926. DYNMOGA has a value of 0.9301 in NMI in period 1. In period 2, this value has improved to 0.9801 but still changes sequentially between 0.9740 and 0.9880 in 3 to 10 time steps. Because DYNMOGA uses the modularity function as the optimization function, we can raise the issue of resolution in the face of these changes.

ESPRA has the highest NMI value in time 1 with 0.9951, and FacetNet has the highest value in time 7 with 0.9655. In Figure 14, the lower error rate is related to our proposed algorithm in all time steps, which, for example, in step 10 was able to achieve the value of 101. In this time step, error rates for other comparable algorithms are 139, 2111, 3899, and 8195 for MSGA, DYNMOGA, ESPRA, and FacetNet, respectively. We observe that in this network, the highest error rate in all time steps is related to the FacetNet algorithm. ESPRA was able to obtain a lower error rate than DYNMOGA in steps 2, 4, and 6. We have already mentioned that the lower the error rate, the higher the accuracy of community detection.

The article "A Multiagent Memetic Optimization Algorithm Based on Temporal Asymptotic Surprise in Complex Networks to Reveal the Structure of the Dynamic Community" was published in 2022. Journal: Comput Intell Neurosci.

Figure 15 shows the performance of our proposed algorithm, DYNMAMA, and the four algorithms MSGA, DYNMOGA, ESPRA, and FacetNet in the merging and splitting section of the LFR database. As you can see, DYNMAMA has been able to detect communities more accurately in obtaining NMI than the other four methods. Also, the presence of the TAS function with the property of breaking the resolution limit in both DYNMAMA and MSGA methods is a better criterion for detecting dynamic communities and can find higher quality communities, which has resulted in an NMI value of either one or almost 1. The NMI values obtained in this section for DYNMAMA ranged from 0.9910 to 1 during steps 1 to 10. MSGA ranged from 0.9881 to 0.9980, and DYNMOGA ranged between 0.9423 and 0.9720. The low NMI for DYNMOGA in step 1 indicates the high error rate of this method in this interval, and gradually with increasing the NMI value, this error rate has improved and does not reach values less than 0.9610. ESPRA and FacetNet obtained the highest NMI values at time step 1 with 0.9886 and 0.9651, respectively, and the lowest NMI values at time step 8 and 9 with 0.9301 and 0.9308 values, respectively. ESPRA obtained higher NMI values than DYNMOGA in steps 1 and 6. In other words, it has been able to detect dynamic communities with better quality than the DYNMOGA method in these two time steps. In Figure 15, the lower error rate is related to our proposed algorithm in all time steps, which, for example, in step 2 was able to achieve the value of 98. The error rates for other comparable algorithms in this time step are 129, 3951, 11151, and 8199 for MSGA, DYNMOGA, ESPRA, and FacetNet, respectively. We observe that DYNMOGA has the highest error rate in time step 1. Also, ESPRA has a higher error rate than FacetNet in steps 2 and 3.

Figure 16 shows a comparison between our proposed method, DYNMAMA, and the four algorithms in obtaining the NMI value for the hidden part of the LFR data set, which still shows the superiority of the DYNMAMA method over the other four methods. NMI values ranged from 0.9988 to 1 for DYNMAMA, 0.9901 to 1 for MSGA, and 0.9520 to 0.9810 for DYNMOGA during steps 1 to 10. But we are still of the opinion that these evolutionary algorithms have always been able to keep the NMI value in the very close range of 1 and always discover higher quality communities. Still, in comparing TAS and modularity evaluation functions, this advantage with TAS is always preserved. Existence of split and merge operators in MSGA, the presence of multiobjective structure using genetic algorithm in DYNMOGA, and the existence of local search and multiagent structure in DYNMAMA have led to this process of improving dynamic communities with higher accuracy and quality. The highest NMI values obtained by ESPRA and FacetNet methods are in steps 1 and 4, respectively, with 0.9881 and 0.9789. In steps 1, 2, and 7, the ESPRA method obtained higher values than the DYNMOGA method. In Figure 16, the lower error rate is related to our proposed algorithm in all time steps, which, for example, in time step 4 was able to achieve the value of 199. The error rates for other comparable algorithms in this time step are 232, 3251, 5741, and 13700 for MSGA, DYNMOGA, ESPRA, and FacetNet, respectively. We see that the highest error rate in time step 1 is related to DYNMOGA and FacetNet algorithms with values of 9451 and 16300.

The article "A Multiagent Memetic Optimization Algorithm Based on Temporal Asymptotic Surprise in Complex Networks to Reveal the Structure of the Dynamic Community" was published in 2022. Journal: Comput Intell Neurosci.

We mentioned earlier that in our proposed algorithm, DYNMAMA and the MSGA algorithm we used for comparison both use the temporal asymptotical surprise (TAS) evaluation function in their optimization. In the following, we show the experimental results on four parts of the LFR data set, which shows the value obtained by the TAS function by both methods and states which way was able to get the higher TAS value.  Figure 17 shows the performance of these algorithms in the birth and death network for the TAS value. As shown in Figure 17, for the LFR network of the birth and death section, the TAS value obtained in our proposed algorithm, DYNMAMA, has increased compared to the MSGA. In time step 1, the value of TAS is equal for both algorithms, but from time step 2 onward, we encounter an increase in the amount of TAS obtained by DYNMAMA. For example, in time step 3, the TAS value of the DYNMAMA method is equal to 2.7845*e* + 03, and for the MSGA method, it is equal to 2.6436*e* + 03. In time stages of 7 to 10, the value of TAS for both ways is close to each other. The evolutionary structure in both methods has improved the value of TAS. However, this advantage is still with the DYNMAMA algorithm until the time step of 10.  Figure 18 shows the performance changes of these algorithms in the expansion and contraction network of the LFR data set. In this section, the closeness of the answers can still be seen, but the superiority in obtaining a higher TAS for the DYNMAMA method has been maintained from time two onward. As we can see in Figure 19, for the LFR network of the merge and split section, the NMI value obtained in our first proposed method, DYNMAMA, has increased compared to the comparison method. In this section, too, DYNMAMA has maintained its superiority in achieving higher TAS values. For example, in step 2, a value of 2.4971*e* + 03 is obtained for our proposed algorithm. A value of 2.2919*e* + 03 is accepted for the MSGA algorithm.

The article "A Multiagent Memetic Optimization Algorithm Based on Temporal Asymptotic Surprise in Complex Networks to Reveal the Structure of the Dynamic Community" was published in 2022. Journal: Comput Intell Neurosci.

Figure 20 shows the performance comparison between these algorithms in the hidden network.

As we can see, for the LFR network of the hide section, the TAS value obtained in our proposed method, DYNMAMA, has increased compared to the MSGA method in time steps 10.

For example, in step 3, a value of 2.7960*e* + 03 is obtained for our proposed algorithm. A value of 2.6510*e* + 03 is obtained for the MSGA algorithm. In step 6, we received a value of 3.3562*e* + 03 for our proposed algorithm. We got a value of 3.2778*e* + 03 for the MSGA algorithm. According to the results obtained in the LFR data set, we can say that our proposed algorithm, DYNMAMA, has been able to perform better in dynamic community detection than MSGA and increase the values of the TAS parameter and NMI value, which indicates the effectiveness of the proposed algorithm.

As we can see in the figures above, DYNMAMA performs better than other algorithms on all networks. Under the same number of evaluations, DYNMAMA can quickly converge to optimum mode with good stability. DYNMAMA can achieve the best-known results better than MSGA and DYNMOGA. DYNMAMA can converge optimally with a small number of evaluations. Having a local search improves the algorithm. The poor scores of genetic algorithms do not converge in a limited number of iterations at each time step. At the same time, the presence of integration and division operators leads to convergence.

### 6.4. Convergence of the Algorithm

We compare the proposed algorithm convergence with other algorithms in this subsection. The convergence graph shows the mean error performance of the best solution over the total runs. The output results are shown in Figure 21. As shown, the proposed algorithm in each repetition achieves better results.

### 6.5. Statistical Analysis

We compare the results of the proposed DYNMAMA algorithm using ANOVA (ANalysis of VAriance) with other algorithms to ensure the statistical results. ANOVA is a statistical test to determine the difference between the meanings of two or more independent statistical populations. In other words, the analysis technique of variance is used to compare two or more groups to investigate whether they are significantly different. ANOVA compares the variance of the between groups with the variance of the within groups. If their variance is not significantly high, the average group may be equal. Tables 5 and 6 present the ANOVA test results for our proposed algorithm compared to other algorithms, including MSGA, DYNMOGA, and ESPRA.

The article "A Multiagent Memetic Optimization Algorithm Based on Temporal Asymptotic Surprise in Complex Networks to Reveal the Structure of the Dynamic Community" was published in 2022. Journal: Comput Intell Neurosci.

Analysis of variance can be used as a method to test the hypothesis of comparing the mean between several independent communities. One of the indicators that can be used to express the characteristics of communities can be the mean. By comparing the mean and detecting their equality or inequality among communities, one can vote for them to be the same or different. Therefore, if one of the means is different from the others, we find that communities are not the same. The test hypotheses for comparing the mean *k* of a community are shown in the following equation:

(9) $$\begin{array}{c} H0:\mu 1=\mu 2=\ldots =\mu k,\\ H1:\text{There are some }\mu^{\prime }\text{s not equal with others.} \end{array}$$

Here, the opposite hypothesis, or  *H*_1_, states that at least one of the means is different from the others, and that the null hypothesis is true, indicating that the means are equal to each other. We see that the *p*− value or sig is less than 0.05. In addition, Figure 22 shows the stability of the compared algorithms in achieving coverage. All algorithms run 20 times independently, and our proposed algorithm has excellent performance in creating full coverage.

## 7. Discussion and Future Work

This paper describes an optimization method based on memetic algorithms and multiagent systems in complex networks to reveal a dynamic community structure. Experiments on the networks used show that our process works well to obtain optimal values. We were able to get good results in the TAS fitness function and the NMI evaluation criterion, which can be found in Tables 3 and 4, and see Figures 11to 20, which show that the answers to the proposed idea are better than the methods compared. In future work, we can combine other evolutionary algorithms with multiagent systems and introduce robust structures to recognize the structure of dynamic communities and increase the strength of this type of network against possible attacks. Let us examine whether combining other evolutionary algorithms with multisystems can create a robust, consistent, and efficient structure for large-scale dynamic networks. The multiagent memetic optimization algorithm proposed in this paper can also solve other optimization problems to improve results and increase efficiency. The output of this community structure detection algorithm can be used in the following cases: recommender systems (people in a community usually have the same interests and tastes, and we can use this to make suggestions in recommender systems), graph visualization tools (communities are usually detected in very large diagrams, and each community is represented by a node that represents all members of that community), link prediction (given that members of a community have many structural similarities, they are more likely to make connections between members of a community in the future), and improved search engines (community detection can also be used in thematic clustering of websites, and this helps to improve the performance of search engines significantly). The above are just a limited number of practical purposes for detecting community structure by our proposed algorithm. In the future, we will generalize our proposed method to weighted and directed networks that exist in large numbers in real life.

The article "A Multiagent Memetic Optimization Algorithm Based on Temporal Asymptotic Surprise in Complex Networks to Reveal the Structure of the Dynamic Community" was published in 2022. Journal: Comput Intell Neurosci.

## 8. Conclusions

One of the most critical issues recently raised in the structure of complex networks is the discovery of communities that change over time, i.e., dynamic communities. Changes in internal links are recorded over time, and it is possible to change the network structure to trace at different time stages. This paper proposes a multiagent optimization memetic algorithm in complex networks to detect dynamic communities in unweighted and undirected complex networks and calls it DYNMAMA (dynamic multiagent memetic algorithm). We can combine multiagent systems and evolutionary algorithms to create new algorithms to solve optimization problems that lead to convergence to optimal global solutions. This convergence occurs at high speed. We, in this paper, use temporal asymptotic surprise (TAS) as an algorithm evaluation function. The temporal asymptotic surprise criterion has a higher resolution than the modularity criterion, breaking the resolution limit. We can obtain a more precise and clear network community structure by maximizing it. TAS can accurately measure the quality of partitions on the dynamic network at a low cost. We also used the NMI to evaluate the quality and accuracy of the dynamic communities received. The goal is to find the optimal community structure. The results of experiments on the real-world Enron email networks and LFR networks show that our proposed algorithm has been able to achieve more efficiency and better answers than the four well-known algorithms for detecting dynamic communities in complex networks. DYNMAMA can handle networks with different densities of edges beside communities by turning the parameter *μ* in LFR networks. Moreover, DYNMAMA has good stability according to the standard deviations and can handle large-scale networks with 1000 nodes. Our proposed algorithm in all time steps was able to obtain the lowest error rate compared to other algorithms, which shows that our proposed algorithm can detect communities with higher accuracy and quality.

The article "A Multiagent Memetic Optimization Algorithm Based on Temporal Asymptotic Surprise in Complex Networks to Reveal the Structure of the Dynamic Community" was published in 2022. Journal: Comput Intell Neurosci.

## Figures and Tables

**Figure 1:** Some examples of community detection methods in dynamic networks.

**Figure 2:** Dense communication of members of a community with each other.

**Figure 3:** Operations in dynamic communities [53].

**Figure 4:** Time-varying community structure.

**Figure 5:** Community evolution in a dynamic network.

**Figure 6:** The structure of an agent.

**Figure 7:** Proposed algorithm (DYNMAMA) parameters.

**Figure 8:** The locus-based representation of an individual. (a) The main structure of the graph; (b) an example of a possible chromosome; (c) structure of communities.

**Figure 9:** The neighborhood of an agent.

**Figure 10:** Flowchart of DYNMAMA.

**Figure 11:** Compare NMI (a) and error rate (b) values in the Enron email network.

**Figure 12:** Compare the Enron email network's TAS values between DYNMAMA and MSGA.

**Figure 13:** Compare NMI (a) and error rate (b) values in the birth and death from the LFR network.

**Figure 14:** Compare NMI (a) and error rate (b) values in the expansion and contraction of the LFR network.

**Figure 15:** Compare NMI (a) and error rate (b) values in the merging and splitting from the LFR network.

**Figure 16:** Compare NMI (a) and error rate (b) values in the hide from the LFR network.

**Figure 17:** Compare TAS values between DYNMAMA and MSGA in the birth and death from the LFR network.

**Figure 18:** Compare TAS values between DYNMAMA and MSGA in the expansion and contraction of the LFR network.

**Figure 19:** Compare TAS values between DYNMAMA and MSGA in the merge and split from the LFR network.

**Figure 20:** Compare TAS values between DYNMAMA and MSGA in the hide from the LFR network.

**Figure 21:** Convergence result of the proposed algorithm compared with the other algorithms in the Enron email network.

**Figure 22:** Stability analysis on the branch coverage.

**Algorithm 1:** DYNMAMA.

**Table 1:** A few examples of memetic algorithms in community detection.

Types of memetic algorithms in community detection		
References	Crossover method	Mutation method
Gong et al. [35]	Two-way X	Neighbor
Zalik and Zalik [36]	X-based modularity and community size	Neighbor
Haque et al. [37]	Add random vertices X	Delete random node
Naeni et al. [38]	Modularity-based X	Adaptive
Wu and Pan [39]	One-way X	Neighbor
Mu et al. [40]	One-way X	One neighbor point
Wang et al. [41]	Uniform X	One point
Ma et al. [42]	Two-way X	Neighbor
Gach and Hao [43]	Priority-based X	—
Gong et al. [44]	—	Neighbor label

The article "A Multiagent Memetic Optimization Algorithm Based on Temporal Asymptotic Surprise in Complex Networks to Reveal the Structure of the Dynamic Community" was published in 2022. Journal: Comput Intell Neurosci.

**Table 2:** Parameter setting.

Parameter	*N*_*s*_	*Ps*	*P*_*b*_	*P*_*a*_	Z_size_
Description	The number of generations	The probability of choosing for hybrid neighborhood crossover operator	Mutation probability	Crossover probability	Population size
Value	500	0.5	0.7	0.7	100

**Table 3:** TAS value for DYNMAMA and MSGA in Enron email network.

				DYNMAMA		MSGA		DYNMOGA	
Time steps	|*V*|	|*E*|	|*E*^*∗*^|	TAS	|*C*|_*D*1_	TAS	|*C*|_*M*_	*Q*	|*C*|_*D*2_
1	91	963	151	173.271	11	169.561	10	0.5219	7
2	95	991	186	179.563	12	178.376	11	0.5348	9
3	90	1431	193	183.112	16	181.593	13	0.5711	11
4	118	1209	245	217.413	13	205.841	14	0.4932	10
5	126	3027	304	223.712	19	218.623	14	0.5984	11
6	108	5129	450	258.903	16	221.179	13	0.6011	11
**7**	124	6698	604	261.015	12	223.602	10	0.5885	9
8	143	6003	864	289.438	17	248.082	14	0.5293	12
9	140	20107	1222	338.517	13	313.977	13	0.5270	9
10	118	6501	614	352.996	12	335.756	11	0.4314	11
11	139	5141	371	353.478	13	341.237	11	0.4993	10
12	117	1657	482	376.025	14	329.668	13	0.5175	9

**Table 4:** The communities detected by DYNMAMA at third and fourth time steps for Enron email network.

Time step: 3		Time step: 4	
Comm. no.	Members	Comm. no.	Members
1	1, 2, 6, 18, 22, 30, 31, 40, 49, 75	1	1, 2, 4, 5, 6, 9, 15, 20, 21, 22, 26, 27, 29, 32, 37, 38, 43, 44, 45, 46, 47, 48, 49, 50, 56, 57, 58, 60, 68, 69, 70, 71, 73, 75, 114
2	3, 9, 21, 23, 36, 42, 45, 55, 122	2	3, 12, 31, 33, 51, 61, 63, 64, 66, 77, 78, 122
3	4, 13, 19, 28, 32, 33, 39, 47, 48, 52, 53	3	7, 11, 53, 74, 118
4	5, 10, 17, 29, 147	4	8, 10, 18, 41, 72, 137
5	7, 12, 51, 137	5	13, 14, 25, 55, 147
6	8, 38, 118	6	16
7	11, 16, 54, 129	7	17, 42, 111
8	14, 27, 46, 50, 151	8	19, 23, 28, 39, 40, 52, 67, 151
9	15, 37, 67	9	24, 34, 76, 129
10	20, 107	10	30, 36, 65, 107
11	24, 125	11	35, 125
12	25, 26, 34, 35, 114	12	54, 62, 150
13	41, 81	13	59, 81
14	43, 150		
15	44, 61		
16	56, 66		

**Table 5:** The ANOVA test for DYNMAMA, MSGA, DYNMOGA, and ESPRA at the 0.05 significant level.

Enron email network	Sum of squares	*df*	Mean square	*F*	Sig.
Between groups	0.715	3	0.238	87.293	0.000
Within groups	0.207	76	0.003		
Total	0.922	79			

**Table 6:** Parameters of descriptive statistical part of ANOVA test for DYNMAMA, MSGA, DYNMOGA, and ESPRA.

Enron email network		*N*	Mean	Std. deviation	Std. error	95% confidence interval for mean		Minimum	Maximum		Between-component variance
						Lower bound	Upper bound				
DYNMAMA		20	0.8379	0.04228	0.00945	0.8182	0.8577	0.76	0.91		
MSGA		20	0.7968	0.04742	0.01060	0.7746	0.8190	0.72	0.89		
DYNMOGA		20	0.7399	0.06053	0.01353	0.7116	0.7682	0.62	0.84		
ESPRA		20	0.5886	0.05670	0.01268	0.5621	0.6152	0.49	0.65		
Total		80	0.7408	0.10803	0.01208	0.7168	0.7649	0.49	0.91		
Model	Fixed effects			0.05224	0.00584	0.7292	0.7524				
	Random effects				0.05457	0.5672	0.9145			0.01177	

The article "A Multiagent Memetic Optimization Algorithm Based on Temporal Asymptotic Surprise in Complex Networks to Reveal the Structure of the Dynamic Community" was published in 2022. Journal: Comput Intell Neurosci.

## Data Availability

Data used in this research are publicly available. The [Real World Network: Enron Email] data and the [Synthetic Network: LFR] data used to support the findings of this study are available at [http:// snap.stanford.edu/data (Stanford Large Network Dataset Collection)], [https://west.uni-koblenz.de/konect], [https://networkrepository.com (Network Repository)], and [http://staff.icar.cnr.it/pizzuti/codes.html]. These prior studies (and datasets) are cited as references at relevant places within the text [3, 4].
